The article "Contrast-Enhanced Ultrasound in the Bladder: Critical Features to Differentiate Occupied Lesions" was published in 2021. Journal: Comput Math Methods Med.

# Contrast-Enhanced Ultrasound in the Bladder: Critical Features to Differentiate Occupied Lesions

**DOI:** 10.1155/2021/1047948

**Published:** 2021-10-12

**Authors:** Qiping Liu, Huiling Gong, Hui Zhu, Chunyan Yuan, Bin Hu

**Affiliations:** ^1^Department of Ultrasound, Minhang Hospital, Fudan University, Shanghai 201199, China; ^2^Department of Pathology, Minhang Hospital, Fudan University, Shanghai 201199, China

## Abstract

**Objective:**

To study the clinical diagnostic value of contrast-enhanced ultrasound (CEUS) in bladder occupied lesions.

**Methods:**

38 cases of conventional-ultrasound-found bladder occupied lesions did color Doppler flow imaging (CDFI) and CEUS checks. By comparing the difference between two types of blood flow imaging technologies in displaying the flow of bladder occupied lesions and observing the perfusion modes of contrast agents to enter lesions, the perfusion characteristics of CEUS were analyzed. Finally, they were contrasted with the surgical pathology results.

**Results:**

Of all the 38 cases, there were 51 bladder occupied lesions, including 43 bladder malignant tumors, 2 bladder inverted papillomas, and 6 glandular cystitis lesions. The blood flow display rate of bladder occupied lesions was 100% using CEUS. Apparently, it was higher than that of CDFI (62.7%), and the result of these showed a statistically significant difference (*P* < 0.05). Using CEUS, 46 malignant lesions and 5 glandular cystitis lesions were indicated, and the diagnostic accuracy rate was 86.3%.

**Conclusion:**

CEUS can improve the blood flow display rate of bladder occupied lesions, and it can also observe the real-time blood flow of these lesions. It can help judge their nature and has a higher clinical value in differentiating the benign from the malignant.

## 1. Introduction

Bladder cancer is the most common malignant tumor in the genitourinary system, and its morbidity and mortality rank the first among male genitourinary tumors in China [1]. As it is convenient, nonradioactive, etc., ultrasonography has been widely used in the diagnosis of bladder tumors and has become an important method to differentiate benign bladder masses from malignant ones. CEUS is a new technique used in clinical practice, which can significantly improve the display rate of low-speed blood flow [2]. CEUS involves the application of ultrasound contrast agents (UCAs), microbubbles with a diameter similar to red cells, to obtain enhanced imaging of the parenchymal microvasculature of tissues based on conventional ultrasonography [3]. In this research, 38 cases with 51 bladder occupied lesions confirmed by surgery or cystoscopy in our hospital the past 7 years were analyzed retrospectively. We used CEUS to detect the blood flow of the bladder occupied lesions. Compared with CDFI, the perfusion mode and perfusion characteristics under CEUS were concluded so as to explore the clinical value of CEUS in the diagnosis of bladder occupied lesions.

The article "Contrast-Enhanced Ultrasound in the Bladder: Critical Features to Differentiate Occupied Lesions" was published in 2021. Journal: Comput Math Methods Med.

## 2. Material and Methods

### 2.1. Patient Population

Collecting bladder occupied lesion cases during August 2013 and November in 2020, which were detected by routine ultrasound examination in our hospital, we had got 38 patients with 51 lesions totally. There were 32 cases with a single lesion, 5 cases with 2 lesions, and 1 case with 9 lesions. Among the patients, 34 male cases got 39 lesions and 4 female cases got 12 lesions. They aged from 32 to 91 years old, 63 years old on average. The size of lesions was 68 × 62 × 56 mm maximum and 6 × 5 × 7 mm minimum. CDFI and CEUS were all performed.

### 2.2. Imaging Techniques

Aplio 500 (Canon, Japan) and Aplio i900 (Canon, Japan) ultrasonic scanners equipped with CDFI and CEUS imaging software were used for an ultrasound examination. Before scanning, the patient was asked to distend the bladder moderately and lay supine on couch. First, a conventional ultrasound scanning, which is focusing on the observation of the location, size, number, morphology, echo, and boundary of the lesions, was performed. After that, CDFI was helped to observe the distribution of blood flow inside and around the lesions (Figure 1). When all the procedures above had been completed, CEUS started. The contrast agent, SonoVue, mixed with 5 mL of normal saline (NS) was preprepared. After windowing the best image of the lesion, 1.6-1.8 mL of the extracted mixture was injected rapidly through the cubital vein, followed by 5 mL of NS, and a timer was set simultaneously. Real-time images were observed continuously for 3-5 mins and archived for offline analysis, including dynamical observation of the changing trend of the contrast agent and a summary of the perfusion pattern of contrast agent in terms of time and echo intensity. To review the playback clips, 2~3 experienced senior sonographers were required. Finally, the medical history and pathological data were followed up for comparative analysis [4].

### 2.3. Statistical Analysis

All statistical analyses were performed by SPSS version 19.0 (SPSS, Inc, Chicago, IL). The chi-square test was used to compare the enumeration data. A *P* value of 0.05 or less was considered statistically significant.

## 3. Results

All the pathology results of bladder occupied lesions were obtained using cystoscopy or transurethral resection of bladder tumor. Of all the 51 lesions in 38 cases, there were 6 glandular cystitis lesions, 2 bladder inverted papillomas, and 43 malignant bladder tumors, including 41 urothelial carcinomas, 1 bladder metastasis of colorectal cancer, and 1 bladder metastasis of prostate cancer.

The article "Contrast-Enhanced Ultrasound in the Bladder: Critical Features to Differentiate Occupied Lesions" was published in 2021. Journal: Comput Math Methods Med.

### 3.1. Internal Blood Flow Showing in the Bladder Mass concerning CDFI and CEUS

Different sizes of bladder masses showed different internal blood flows (Table 1). The display rate of CDFI was 62.7% (32/51), and that of CEUS was 100% (51/51). In general, the color Doppler flow rate of CEUS was higher than that of CDFI, and it was statistically significant (*P* < 0.05).

### 3.2. Manifestation of CEUS

Under 2-dimensional ultrasound, bladder occupied lesions are cauliflower-like or papillary medium-echo mass, hypoechoic mass, and other masses, which are protruding into the bladder cavity and not moving when the body position is changed. Under color Doppler ultrasound, part of them shows stellate or rich blood flow signals. Under CEUS, the ultrasound contrast agents (UCAs) were observed being fast-into and slowly out of the 44 lesions and hyperenhanced (Figure 2), which were indicating bladder malignancy. Pathological results showed 37 lesions of urothelial carcinomas, 1 bladder metastasis of colorectal cancer, 1 bladder metastasis of prostate cancer, 2 bladder inverted papillomas, and 3 glandular cystitis lesions. The UCA was observed being fast-in and slowly out of the lesion and isoenhanced in one lesion and a little perfusion in another lesion. When CEUS indicated these 2 lesions of bladder malignancy, both the pathological results were urothelial carcinomas. The UCAs were observed being slowly in and homogeneously out and isoenhanced in 2 lesions (Figure 3), homogeneously in and homogeneously out and isoenhanced in one lesion. The CEUS indicated glandular cystitis lesions, which also fit with the pathological results. The UCAs were observed being homogeneously in and homogeneously out and hyperenhanced in 2 lesions, which were considered glandular cystitis lesions. But the pathological results actually were urothelial carcinomas. The coincidence rate of CEUS in qualitative diagnosis of benign and malignant bladder tumors was 86.3% (44/51).

## 4. Discussion

Bladder tumors are the most common tumors in urinary system, of which transitional epithelial tumors account for more than 90%. The age of onset was mostly from 50 to 70 years old, and the incidence rate in males was significantly higher than that in females; the proportion was about 4 to 1. Hematuria is the most common and earliest symptom of bladder cancer, and frequent urination, urgent urination, and dysuria are mostly late manifestations of bladder tumors [5]. At present, the main methods for diagnosing bladder occupied lesions include ultrasound, computed tomography (CT), and magnetic resonance image (MRI) [6–8]. As color Doppler ultrasound can detect lesions as small as 5 mm, early detection and early treatment can be achieved, which is of great significance for the observation of pelvic lymph node metastasis and lesion invasion in patients with bladder cancer [9]. Due to the fine blood vessels in the normal bladder, it is difficult to display under CDFI. After the bladder malignant tumor occurred, it is possible to analyze the blood supply inside tumors under CDFI [10]. Because rapid growth of the tumor requires independent arterial blood supply, on the one hand, there are abundant new blood vessels on the other hand. CDFI is of great value for the display of blood supply in bladder tumors and the determination of malignancy [11]. Some studies suggest that CDFI can only display blood vessels no finer than 1-2 mm and can do nothing with finer ones [12]. CEUS is a new technique applied in clinical practice in recent years, which can significantly improve the display rate of low-speed blood flow so as to evaluate the blood perfusion characteristics of organs and lesions. With the help of CEUS, it is possible to show the nourishing vessels of tumors, to reflect the real blood supply characteristics of tumors, and to judge the nature of tumors [13–15]. Compared with CT and MRT, CEUS offers the advantage of nonionizing radiation different from CT, and CEUS is much wider availability and much more cost-effective than MRI. In this study, there were 38 cases with 51 lesions. The display rate of CDFI was 62.7% while that of CEUS was 100%, which was significantly higher.

The article "Contrast-Enhanced Ultrasound in the Bladder: Critical Features to Differentiate Occupied Lesions" was published in 2021. Journal: Comput Math Methods Med.

CEUS is a new technique developed in recent years that can objectively reflect tissue perfusion. It uses microbubble contrast agent to show the blood flow distribution in and around the lesion by developing fine blood vessels and tumor nourishing vessels. Sonovue, a new ultrasound contrast agent, is a blood pool tracer that never leaves the blood vessel and can be used for real-time dynamic observation of microcirculation perfusion [16]. Bladder malignant tumors get a fast-into and slowly out and hyperenhanced imaging mode in contrast with their own bladder wall tissue, whereas benign lesions get isoenhancement and hypoenhancement and nonenhancement imaging modes. It can not only differentiate malignant lesions from benign ones but also greatly improve the qualitative diagnostic accuracy of bladder occupied lesions under CEUS, depending on different UCA perfusion strength and enhancement modes [17]. In this study, the diagnostic accuracy of CEUS was 86.3%. In addition, CEUS combined with grayscale (US) ultrasonography and monochromatic superb microvascular imaging (mSMI) can improve diagnostic efficiency for bladder occupied lesions. Through CEUS, we can observe the blood flow of bladder tumors in real time, which is helpful to judge the nature of tumors and provide a basis for the differential diagnosis of benign and malignant tumors [18]. In this study, 2 bladder inverted papilloma cases were misdiagnosed as bladder malignancy, so that it may be somewhat difficult to distinguish this disease from bladder malignancy [19]. A bladder inverted papilloma is a urinary epithelial benign tumor. Most of them have regular shapes, which look pedunculated and papillary, and smooth surfaces. They show slightly strong echoic or hyperechoic, and there is homogeneous inner echo in most cases and inner spotted strong echo in part of cases. Some masses get a strong echoic outline and hypoechoic inside. Some scholars think that all above are the characteristic ultrasonographic manifestation of bladder inverted papillomas different from bladder cancers [20].

The article "Contrast-Enhanced Ultrasound in the Bladder: Critical Features to Differentiate Occupied Lesions" was published in 2021. Journal: Comput Math Methods Med.

In this study, 3 cases of glandular cystitis were misdiagnosed as bladder malignant tumors under CEUS, because of the contrast findings, who showed fast-in and slowly out imaging mode and hyperenhanced in tumors compared with their bladder wall, which was similar to that of bladder malignant tumors. It suggested that the blood supply of glandular cystitis could also be extremely rich, so more attention should be paid to the differential diagnosis [21]. However, if a small cystic anechoic area is seen in the lesion, it is the characteristic manifestation of glandular cystitis [22].

A bladder mass also needs to be differentiated from bladder blood clot, umbiliculopathy and other diseases. Intrabladder blood clots float when patients turn over, but bladder masses do not [23]. A bladder mass shows blood supply under CDFI or CEUS, while an intrabladder blood clot does not show any blood supply. Ultrasonography of umbiliculopathy shows a hypoechoic mass convex from the anterior wall of the bladder to the outside of the lumen [24], while a bladder mass is convex to the inside, which is more likely to occur in the trigonum and lateral wall of the bladder. Cystoscopy is feasible to confirm the diagnosis.

There are some disadvantages in this study, including a small sample size, especially fewer cases of benign bladder tumors, lack of further research in the degree, and stage of bladder tumor invasion. We will try our best to make up for the above deficiencies in our future work and research.

In conclusion, as a new technique, CEUS can reflect the blood supply inside the tumor and significantly improve the blood flow display rate of bladder occupied lesions. Meanwhile, CEUS has high clinical application value in the diagnosis and differential diagnosis of benign and malignant bladder occupied lesions according to its contrast mode.

The article "Contrast-Enhanced Ultrasound in the Bladder: Critical Features to Differentiate Occupied Lesions" was published in 2021. Journal: Comput Math Methods Med.

## Figures and Tables

**Figure 1:** The manifestation of the bladder occupied lesion under CDFI. (a) No inner blood flow in glandular cystitis lesion; (b) no inner blood flow in bladder malignant tumors.

**Figure 2:** The manifestation of the bladder malignant tumor under CEUS. (a) Fast-in mode; (b) hyperenhancement at its peak time; (c) slowly out mode.

**Figure 3:** The manifestation of the glandular cystitis under CEUS. (a) Slowly in mode; (b) isoenhancement at its peak time; (c) homogeneously out mode.

**Table 1:** Internal blood flow showing in the bladder mass concerning CDFI and CEUS.

Diameter of masses	N	CDFI		CEUS		*P*
		+	-	+	-	
≤2.0 cm	19	6	13	19	0	0.00001
>2.0 cm	32	26	6	32	0	0.01008
	51	32	19	51	0	<0.00001

## Data Availability

The datasets used and/or analyzed during the current study are available from the corresponding author on reasonable request.
